RETRACTED

# *Astragali radix*: could it be an adjuvant for oxaliplatin-induced neuropathy?

**DOI:** 10.1038/srep42021

**Published:** 2017-02-10

**Authors:** Lorenzo Di Cesare Mannelli, Alessandra Pacini, Laura Micheli, Angelo Pietro Femia, Mario Maresca, Matteo Zanardelli, Alfredo Vannacci, Eugenia Gallo, Anna Rita Bilia, Giovanna Caderni, Fabio Firenzuoli, Alessandro Mugelli, Carla Ghelardini

**Affiliations:** 1 Dept. of Neuroscience, Psychology, Drug Research and Children’s Health - NEUROFARBA - Pharmacology and Toxicology Section, Florence, Italy; 2 Dept. of Experimental and Clinical Medicine - DECM - Section of Anatomy and Histology, University of Florence, Florence, Italy; 3 Department of Chemistry, University of Florence, Florence, Italy

## Abstract

Neurotoxicity is a major side effect of platinum derivatives both during and after treatment. In the absence of effective pharmacological compounds, the opportunity to identify safe adjuvant treatments among medicinal plants seems appropriate. *Astragali radix* is an adaptogenic herbal product recently analyzed in platinum-treated cancer patients. With the aim of evaluating the anti-neuropathic profile of Astragali radix, a previously characterized aqueous (Aqu) and two hydroalcoholic (20%HA and 50%HA) extracts were tested in a rat model of oxaliplatin-induced neuropathy. Repeated administrations significantly reduced oxaliplatin-dependent hypersensitivity with 50%HA, the most effective, fully preventing mechanical and thermal hypersensitivity. *Ex vivo*, 50%HA reduced morphometric and molecular alterations induced by oxaliplatin in peripheral nerve and dorsal-root-ganglia. In the spinal cord and in brain areas, 50%HA significantly decreased activation of microglia and astrocytes. Furthermore, 50%HA prevented the nephro- and hepato-toxicity induced by the anticancer drug. The protective effect of 50%HA did not alter oxaliplatin-induced apoptosis in colon tumors of Pirc rats, an Apc-driven model of colon carcinogenesis. The hydroalcoholic extract (50%HA) of Astragali radix relieves pain and promotes the rescue mechanisms that protect nervous tissue from the damages triggering chronic pain. A safe profile strongly suggests the usefulness of this natural product in oxaliplatin-induced neuropathy.

Oxaliplatin is a third-generation platinum drug, extensively used, in a combination with 5-fluorouracil and leucovorin, for the management of locally advanced and metastatic cancer of the colon or rectum^1^. A major limitation associated with the use of oxaliplatin is represented by its neurotoxicity, which leads to painful neuropathy. Acute symptoms appear shortly after infusion but usually vanish within a week^2^. By contrast, cumulative oxaliplatin administrations cause chronic neuropathy in approximately 50% of patients receiving doses higher than 1000 mg/m^2^ 3,4. Paresthesia, dysesthesia and pain combined with a glove-and-stocking distribution sensory loss are the most common signs of neuropathy development^5^,^6^. During treatment, chemotherapy-induced neuropathy can limit therapeutic options for patients and result in dose reduction. During survival, it might greatly affect the patient’s quality of life^7^.

RETRACTED

The 2014 practical clinical guideline from the American Society of Clinical Oncology states that there are no agents recommended for the prevention of chemotherapy-induced neuropathic pain^8^. No progress has been achieved up to now^9^. High-quality, consistent evidence is insufficient; the best available data support a moderate recommendation for treatment with duloxetine^10^,^11^. Consequently, the prevention or treatment of oxaliplatin-induced neuropathy (as well as other chemotherapy induced neuropathies) is a relevant therapeutic need.

In this context, a scientific approach to the study of medicinal plants may help to identify adjuvant treatments able to reduce the side effects of chemotherapy. Phytotherapy is based on the combined action of a mixture of constituents able to offer a multiple approach to the multi-factorial nature of neuropathy pathogenesis. The bioactivity of crude drugs or vegetal extracts is a summation of antagonistic and/or synergistic effects on bioavailability, cellular transport processes, compound metabolism and pharmacodynamic mechanisms^12^.

Recently, we demonstrated the protective effect of different extracts of Astragali radix in a cellular model of oxaliplatin-induced neurotoxicity^13^. Importantly, none of the tested extracts interfered with the toxicity elicited by oxaliplatin in the human colon adenocarcinoma cell line HT-29.

Astragali radix is one of the important “Qi tonifying” or adaptogenic herbs from the Chinese *materia medica* (recently introduced in the European Pharmacopoeia). It has been prescribed for centuries for general debility, chronic illnesses, and to increase the overall vitality of the system^14^. Current evidence about the combination of *Astragalus* extracts and chemotherapy (in particular with the FOLFOX regimen) highlight a significant improvement in the patient’s quality of life^15^,^16^,^17^,^18^.

The present study is focused on the evaluation of the anti-neuropathic properties of different Astragali radix extracts (aqueous, Aqu, and two hydroalcoholics, 20%HA and 50%HA) in rats subchronically treated with oxaliplatin. The relief of pain hypersensitivity as well as the protective effects on the peripheral and central nervous system were analyzed. Finally, the influence of *Astragalus* on the anticancer properties of oxaliplatin was evaluated in Pirc rats, an Apc-driven model of colon carcinogenesis, measuring oxaliplatin-induced apoptosis in colon tumors as a marker of its therapeutic effect.

RETRACTED

## Results

### Behavioral measurements

On day 21, oxaliplatin administration to Sprague-Dawley rats (2.4 mg kg^−1^ intraperitoneally - i.p. - daily, for 5 consecutive days/week for 3 weeks) altered the sensitivity to both noxious and non-noxious mechanical stimuli. As measured by the Paw pressure test, oxaliplatin treatment lowered the pain threshold in response to a mechanical noxious stimulus, reducing the control value from 66.5 ± 1.9 g to 40.7 ± 1.8 g (Fig. 1A). The treatment with Aqu and 20%HA (300 mg kg^−1^ *per os* - p.o. - daily from the first day in which the chemotherapic compound was injected) reduced the pain behavioral alterations whereas 50%HA (300 mg kg^−1^ daily p.o. following the same protocol) fully prevented the sensitivity to noxious mechanical stimuli (Fig. 1A).

The withdrawal threshold to a non-noxious mechanical stimulus, measured by the electronic Von Frey apparatus, was decreased in oxaliplatin-treated animals (day 21) from 23.7 ± 1.2 g, to 13.8 ± 0.9 g (Fig. 1B). The pro-allodynic effect of oxaliplatin was significantly reduced by Aqu and totally prevented by both 20%HA and 50%HA (Fig. 1B).

The response to a non-noxious thermal stimulus is shown in panel C of Fig. 1. The anticancer agent decreased the licking latency in the Cold plate test from 24.1 ± 1.2 s (vehicle + vehicle) to 16.2 ± 0.8 s (oxaliplatin + vehicle). Administration of 50%HA was the only dose able to significantly reduce oxaliplatin-induced cold hypersensitivity (Fig. 1C).

The above described treatments with Aqu, 20%HA and 50%HA performed on control rats (which did not receive oxaliplatin) did not alter the pain threshold evaluated using the Paw pressure, Von Frey and Cold plate tests (Fig. 1A,B and C).

To better evaluate the pain relief profile of 50%HA, the extract was administered p.o. daily (subchronic; from the first day in which oxaliplatin was injected) at 3 different dosages, 30, 100 and 300 mg kg^−1^. On day 21, the pain threshold measurement by the Paw pressure test showed that 50%HA provided a dose-dependent protective effect after repeated treatment (Fig. 2, subchronic). The full efficacy of 50%HA was shown also on day 14, suggesting early beneficial effects (Supplementary Fig. S1). On the contrary, 300 mg kg^−1^ 50%HA acutely administered p.o. on day 21 did not modify the pain threshold decreased by oxaliplatin (Fig. 2, acute).

Once evaluated the activity of the phytocomplex 50%HA, we aimed to enquire the possible efficacy of single fractions of the crude extract. 50%HA was suspended in water and extracted with solvents with increasing polarity (dichloromethane, ethyl acetate, butanol, water). After liophylization we obtained solid products in the following percentage (compared to the quantity of the total extract): 1) dichloromethane fraction, 22%; 2) ethyl acetate fraction, 3%; 3) butanol fraction, 6%; 4) water fraction, 69%. Accordingly, different groups of animals were treated with dosages representing these percentages of the total extract dose (300 mg kg^−1^). In particular, 1) dichloromethane fraction, 66 mg kg^−1^; 2) ethyl acetate fraction, 9 mg kg^−1^; 3) butanol fraction, 18 mg kg^−1^; 4) water fraction, 207 mg kg^−1^. These treatments were compared with effects due to the administration of the mixture of all fractions at the same doses. As shown in the Supplementary Fig. S2, none of the single fractions induced a significant effect whereas the animals that received the co-administration of all the fractions showed a decrease of pain hypersensitivity comparable to that induced by the total crude extract.

RETRACTED

Finally, oxaliplatin negatively influenced motor coordination. The Rota rod test measures the walking time and number of falls in 600 s from a rotating rod. Oxaliplatin-treated animals showed reduced walking time (197.8 ± 24.8 s; Supplementary Fig. S3A) and an increased number of falls (4.4 ± 0.5; Supplementary Fig. S3B) in comparison with control animals (600 s and 0.7 ± 0.3, respectively). Repeated administration of each Astragali radix extract (300 mg kg^−1^ daily p.o. starting from the first day of oxaliplatin injection) restored motor coordination, improved the time spent in equilibrium on the rod and reduced the number of falls (Supplementary Fig. S3B). In the absence of oxaliplatin, repeated treatment with *Astragalus* extracts did not alter motor coordination *per se* (Supplementary Fig. S3A and B).

### p-NF-H expression in the sciatic nerve

Expression level evaluation of the phosphorylated form of the heavy polypeptide of neurofilament (p-NF-H, a major determinant of axonal structure and functionality^19^) in the rat sciatic nerves showed an oxaliplatin-dependent down-regulation (Fig. 3A, oxaliplatin + vehicle) compared to the vehicle control group (Fig. 3A, vehicle + vehicle). Compared to the oxaliplatin group, nerve sections of 50%HA treated rats (Fig. 3A, vehicle + 50%HA) exhibited a p-NF-H increment. The immunolabeling observed in the presence of 50%HA alone (Fig. 3A, vehicle + 50%HA) did not show any significant difference in comparison to control (Fig. 3A, vehicle + vehicle).

RETRACTED

### Histology and morphometry of dorsal root ganglia (DRG)

The features of oxaliplatin-induced neuronopathy have already been reported in detail^19^,^20^,^21^. To summarize, the main pathological changes were found in the nucleolus and the nucleus of the DRG neuronal cells where an increased incidence of multinucleolated cells (Fig. 3B, black arrow in oxaliplatin + vehicle, and striped bar in upper histogram) and nucleolar segregation (Fig. 3B, black arrow in oxaliplatin + 50%HA, and striped bar in lower histogram) were evidenced. On the contrary, the neuronal cytoplasmic involvement was very limited. Quantitative analysis of the multinucleated nuclei (upper histogram) and eccentric nucleoli (lower histogram) in the presence of 50%HA was significantly reduced (Fig. 3B, oxaliplatin + 50%HA and gray bars) compared to oxaliplatin alone.

### ATF-3 expression in L4-L5 DRG

Expression of the activating transcription factor 3 (ATF-3) in DRG is considered a neuronal marker of nerve injury^22^. Immunohistochemistry was used to assess its expression in the presence or in the absence of 50%HA (Fig. 3C). ATF-3-positive cells from 3 non-adjacent transverse sections (10 μm) of L4 and L5 DRG *per* animal (*n* = 6 per group) were counted, and expressed as a percentage of the total number of cells counted in these sections. DRG neurons showed significant ATF-3 expression following oxaliplatin treatment (striped bar), whereas the presence of 50%HA (gray bar) displayed a significant reduction of ATF-3 nuclear immunoreactivity. No differences were observed following 50%HA treatment alone (white bar) in comparison with control (black bar). Representative photomicrographs show the 50%HA protective nuclear effect (oxaliplatin + 50%HA) compared to oxaliplatin treatment (oxaliplatin + vehicle, black arrows).

### Spinal and cerebral glial analysis

As we have previously reported^19^, a 3 week oxaliplatin treatment is associated with a numeric and morphological astrocyte boost within the spinal cord, where the increase in the cell body size denotes their typical activated state (Fig. 4A, oxaliplatin + vehicle, see insert for morphological details). On the contrary, microglia did not undergo any of the above modifications (data not shown). Treatment with 50%HA resulted in a numerical reduction of astrocytes within the dorsal horns as demonstrated by immunohistochemistry for the astrocytic marker Glial Fibrillary Acidic Protein (GFAP) (Fig. 4A, oxaliplatin + 50%HA). Rats that received only 50%HA (vehicle + 50%HA) were indistinguishable from control rats (vehicle + vehicle), showing no astrogliosis or morphological modifications.

Under the same conditions, we measured the density of astrocytes (GFAP) and microglia (by means of the Iba1 specific marker) in several brain areas known to be active during chronic pain^23^,^24^ and already demonstrated to be involved in cerebral gliosis following oxaliplatin-administration^19^. In all examined areas, our results demonstrated a 50%HA-dependent reduction in the density of both astrocytes and microglia (Fig. 4B and C, gray bars, respectively) in comparison to oxaliplatin-treated rats (striped bars). Rats treated with only 50%HA did not exhibit any differences from control animals (data not shown).

RETRACTED

### Nrf2 and NQO1mRNA levels in the nervous system

To assess the redox profile after treatments, two major cellular antioxidant players were analyzed. Oxaliplatin treatment did not modify the nuclear factor (erythroid-derived 2)-like 2 (Nrf2) mRNA either in the sciatic nerve or in the spinal cord (Supplementary Fig. S4A and C). On the contrary, Nrf2 increased in DRGs, 50%HA significantly prevented this alteration (Supplementary Fig. S4B). 50%HA decreased Nrf2 spinal levels (oxaliplatin + 50%HA) in comparison to control (Supplementary Fig. S4C). Similarly, 50%HA decreased the NAD(P)H dehydrogenase, quinone 1 (NQO1) (oxaliplatin + 50%HA) in DRGs in comparison to control (Supplementary Fig. S4B). Oxaliplatin reduced NQO1 levels in the spinal cord, 50%HA was not effective (Supplementary Fig. S4C).

### Hepatic and renal histopathological features

Given the neuroprotective properties of 50%HA, we examined its potential protective effects against hepatic and renal toxicity induced by oxaliplatin treatment. The macroscopic liver appearance of the vehicle + vehicle-treated animals appeared normal without any alterations in terms of shape, dimension, hue or solidity (data not shown). The microscopic examination of liver sections from the control rats showed a normal lobular pattern, hepatic cells with well-preserved cytoplasm, prominent nucleus, nucleolus and a well-defined central vein. There was no sign of inflammation or fatty change (Fig. 5A, vehicle + vehicle). In animals administered with oxaliplatin alone, liver sections showed marked congested central veins and sinusoids, multifocal areas of necrosis, increased fatty deposits (insert in Fig. 5A, oxaliplatin + vehicle, black arrow) and the presence of inflammatory cells with granular swelling (insert in Fig. 5A, oxaliplatin + vehicle, black arrowhead). Treatment with 50%HA resulted in a considerable reduction in necrotic areas, with disappearance of inflammatory infiltrates and a remarkable improvement in the macrovesicular fatty changes of the hepatic parenchyma (Fig. 5A, oxaliplatin + 50%HA). Figure 5A (vehicle + 50%HA) shows that there was no sign of alterations in animals administered with 50%HA alone.

RETRACTED

Figure 5B (oxaliplatin + vehicle) shows representative hematoxylin-eosin stained sections demonstrating the glomerulopathy with cytopathic changes developed by oxaliplatin-treated kidney. In particular, glomerular alterations consisted of mesangial expansion (Fig. 5B left panel, oxaliplatin + vehicle, black arrowhead), glomerular hyalinization, Bowman’s space expansion (Fig. 5B left panel, oxaliplatin + vehicle, black asterisk) with a coarctation of the entire glomerulus, and Bowman’s capsule basement membrane thickening (Fig. 5B left panel, oxaliplatin + vehicle, black arrow). The administration of 50%HA concurrently with oxaliplatin, exhibited protective effects detectable as less severe glomerular damages and a reversal of the vacuolar degenerative changes of the tubular cells (Fig. 5B, oxaliplatin + 50%HA).

### Apoptosis in tumors and normal mucosa of Pirc rats

To gather information on the possible interference of *Astragalus* with the toxic effect of oxaliplatin in colon tumors, we measured the level of apoptosis in tumors and normal mucosa of Pirc rats with spontaneous tumorigenesis. Oxaliplatin or oxaliplatin + 50%HA was administered to Pirc rats from the eighth to the ninth months of age, when colon tumors had already developed. These animals were more sensitive to the general toxicity of oxaliplatin, showing strong anemia, asthenia and weight loss when treated with 2.4 mg kg^−1^ oxaliplatin daily. For this reason, the treatment was modified to 1.5 mg kg^−1^ i.p. twice weekly for 4 weeks. As shown in Fig. 6A, Pirc rats showed hypersensitivity to mechanical stimuli (Paw pressure test) starting on week 1 (after two injections) with a continual pain threshold decrease over time.

In parallel, another group of animals underwent a 4-week treatment with oxaliplatin (1.5 mg kg^−1^ i.p. twice weekly) and 50%HA (300 mg kg^−1^ p.o. daily starting on the first day of oxaliplatin administration). 50%HA significantly prevented pain development (Fig. 6A). The week 4 was chosen as optimal for neuropathy establishment and duration of 50%HA treatment. On week 4, Pirc rats (9 months old) were sacrificed and apoptosis was evaluated in colon tumors as well as in the apparently normal mucosa. The treatment with 50%HA did not affect the apoptotic index either in the normal mucosa or in the tumors (Fig. 6B), demonstrating that 50%HA did not interfere with oxaliplatin’s pharmacological effect. In agreement with other authors^25^, the level of apoptosis in tumors was significantly higher than that in normal mucosa.

## Discussion

The present data show the anti-neuropathic effects of different Astragali radix extracts in a rat model of oxaliplatin-induced neurotoxicity. In particular, 50%HA controls pain and prevents damage to the peripheral nervous system and the maladaptive changes along the entire nociceptive pathway within the central nervous system.

RETRACTED

Aqu, 20%HA, and 50%HA significantly reduce the pain sensitivity alterations caused by repeated administrations of the platinum derivative. 50%HA is the most effective, fully preventing hypersensitivity to suprathreshold stimulation (hyperalgesia-related measurement) and pain threshold alterations to stimuli that normally do not provoke pain (allodynia-related measurement). Pain relief was observed after a subchronic treatment, suggesting a neuroprotective mechanism against the damages that result in chronic pain. Accordingly, 50%HA prevents morphological derangements in DRGs, a primary target for oxaliplatin neurotoxicity^19^,^26^, as well as the significant increase in ATF-3 expression, a member of the ATF-3/cAMP-responsive element binding protein family considered a selective marker of neuronal damage^19^,^20^,^27^. Moreover, 50%HA prevents the downregulation of the phosphorylated heavy neurofilament, a parameter indicative of latent axonal damage^19^,^28^.

*In vitro*, we recently described the protective characteristics of 50%HA against the toxicity evoked by oxaliplatin in primary astrocytes^13^. Glial cells have been recognized as powerful modulators of pain^29^. The metabolic activation of microglia and astrocytes participates in the maladaptive plasticity of the central nervous system, facilitating nociceptive processes, generating clinical pain hypersensitivity and making neuropathic pain an autonomous disease state^29^.

Despite the limited ability of oxaliplatin to cross the blood brain barrier^30^, we previously observed glial activation induced by oxaliplatin in spinal cord and brain areas differently according to cell type, anatomical region, and treatment time-points^19^. The increased cell density of microglia and astrocytes is strongly related to pain hypersensitivity since the glial inhibitor minocycline and fluorocytrate fully prevent oxaliplatin-evoked pain^21^. The present results reveal an inhibitory effect of 50%HA on microglia and astrocytes (decreasing in the number of both cell types) in the dorsal horn of the spinal cord, in brain areas belonging to the “pain neuromatrix”^31^ and in other brain networks involved in somatosensory, motor, attention and emotional processing^32^. To note, 50%HA seems to be able to modulate glial cells instead of acting as a general depressor of glial functions. The homeostatic properties of the *Astragalus* extract may allow inhibition of glial hyper-reactivity but preserve neuroprotection, a housekeeping role of these cells^33^.

RETRACTED

Several bioactive compounds have been highlighted in the dried root of *Astragalus* such as isoflavonoids (calycosin and formononetin), triterpene saponins (whose major component is represented by Astragaloside IV)^34^, polysaccharides, amino butyric acids and various trace elements^15^,^35^,^36^. The phytochemical characterization of the present extracts reveals the presence of these active compounds, showing similar contents of total saponins in Aqu, 20%HA and 50%HA whereas isoflavones are more concentrated in the hydroalcoholic extracts of Astragali radix rather than in Aqu^13^. Since *Astragalus* flavonoids, saponins and polysaccharides^15^,^36^,^37^ possess considerable activities against oxidative imbalance and oxaliplatin induces oxidative damage relevant for pain sensitivity^38^, the mRNA levels of redox-related molecules are studied in different nervous districts. Nrf2 is an important cellular defense response against oxidative or electrophilic stress^39^, it plays an imperative role in inhibiting oxidative stress via upregulating the Nrf2-driven antioxidants, including mainly heme oxygenase 1 (HO-1), NQO1 and γ-glutamate-cysteine ligase (γ-GCL)^40^. In oxaliplatin-treated animals Nrf2 slightly increases in DRGs whereas NQO1 decreases in the spinal cord. 50%HA reduces both Nrf2 and NQO1 levels in DRGs and spinal cord, suggesting the lack of a direct stimulation of the cellular antioxidant machinery. Nevertheless, because of the neuroprotective profile of 50%HA, less need of physiological antioxidant responses after *Astragalus* administration could be hypothesized. The neuroprotective properties of *Astragalus* root components have been previously described. Formononetin was able to preserve neurons from apoptosis^41^. Astragaloside IV reduced caspase-3 activation, protected fiber demyelination and promoted peripheral nerve regeneration in animal models of neuropathy^42^.

A general restorative property of *Astragalus* extracts has also been reported: anti-hypertensive and immunomodulatory activities^15^ as well as the capability to protect the liver and reduce hyperglycemia^43^. In the present results, histological observations of the liver and kidney also strongly support the hepato- and kidney-protective effect of 50%HA against oxaliplatin-induced organ toxicity.

It is relevant to underline that the efficacy of 50%HA is strongly related to the whole phytocomplex. Aimed to study the role of the different chemical families present in the extract, we have been performed a fractionation by solvents with increasing polarity (dichloromethane, ethyl acetate, butanol and water). The procedure let to the separation of constituents on the basis of their different polarity, namely lipophilic constituents have been solubilized in dichloromethane, the aglycons of saponins and flavonoids and their less polar glycosides in ethyl acetate, saponins and flavonoids glycosides (and all the other polar constituents not completely soluble in water) in butanol. Final water fraction contains only constituents such as simple sugars or polysaccharides. After repeated administrations, none of these fractions show pain relieving properties in oxaliplatin-treated animals. On the contrary, the animals that received the co-administration of all the fractions show a decrease of pain hypersensitivity comparable to that induced by the total crude extract suggesting the synergy of several compounds and validating the traditional phytotherapic approach.

RETRACTED

As regards safety against chemotherapy, the lack of interference of *Astragalus* extract (50%HA) in oxaliplatin-induced caspase-3 activation and cell mortality in the colon cancer cell line HT-29 has been previously reported^13^. In the present study, the possible *Astragalus* interference with the anticancer activity of oxaliplatin was evaluated *in vivo* in Pirc rats, a genetic model of colon cancer. This rat strain harbors a heterozygous mutation in Apc, the key gene in colon carcinogenesis. Accordingly, Pirc rats spontaneously develop tumors in both the small and large intestines, mimicking the human pathology^44^. We used this model to ascertain if 50%HA would impede the chemotherapic effect of oxaliplatin on tumors. Apoptosis was measured in the normal mucosa and tumors, and our results indicate that 50%HA does not interfere with oxaliplatin-induced apoptosis in either tissue, thus suggesting that *Astragalus* does not modify the anticancer efficacy of the platinum derivative.

On the other hand, compelling evidence suggests the usefulness of Astragali radix in cancer treatment. *Astragalus* is included among the specific plants that contribute to tumor response when combined with oxaliplatin-based chemotherapy for colorectal cancer^17^. The combination of Chinese herbal medicine, including Astragali radix, improved the effectiveness of FOLFOX against advanced colon cancer in terms of tumor response rate and one-year survival. Patients also reported fewer adverse effects and experienced better quality of life^16^. A metanalysis of randomized trials concluded that *Astragalus*-based treatment increased the efficacy (by improving survival, tumor response, and performance status) and reduced the toxicity of standard platinum-based treatment in patients affected by advanced non–small-cell lung cancer^45^. Anticancer properties were suggested for Astragaloside IV which exhibited *in vivo* anticancer activity and enhanced immune response^46^. *Astragalus* saponins inhibited proliferation in a human colorectal cancer HT-29 cell line regardless of the p53 status, demonstrating tumor suppressive effects in a nude mice xenograft model and enhancing the cytotoxic effect of 5-FU^47^. Cui *et al*. highlighted the anti-tumoral activity of *Astragalus membranaceus* in counteracting hepatocarcinogenesis in rats^48^. *Astragalus* polysaccharides have demonstrated to have anti-proliferative effects in cell-line studies^49^.

RETRACTED

## Conclusions

Since improved cancer therapy has led to increased life expectancy and cure rates in most types of cancers, the issue of symptom management has begun to play a very important role^6^. Pain is a prominent under-treated symptom in cancer^50^; no effective agents are available for the treatment of chemotherapy-induced neuropathy^8^. The Astragali radix hydroalcoholic extract 50%HA was able to control oxaliplatin-induced pain and prevent alterations in both the peripheral and central nervous system. 50%HA may offer a dual protective approach against etiological factors and resulting maladaptive plasticity without altering the anticancer efficacy of oxaliplatin.

## Methods

### Plant material, sample preparation and analysis

A commercial sample (0.5 kg dry herbal drug) of Astragali radix (Huang Qi) was purchased from Gansu China Shenzhen Green Nature Co. LTD. The Art. No. was 30237, China production lot no. 0061, July 2010. The plant material was comminuted, reduced to a powder form, and used to make the extracts. The decoction (Aqu) was prepared using 5 g of the herbal drug plus 100 mL distilled water and boiled for 4 h on a heating plate (adding water when necessary to maintain a constant volume). After 4 h of boiling, the decoction was cooled down to room temperature on a horizontal shaker to improve the bottom deposition of the solid drug. It was then filtered and centrifuged (5000 rpm, Δt = 10 min, temp. = 20 °C), and after that, the extract was frozen (−24 °C) and lyophilized.

The 20%HA extract was prepared with 5 g of the herbal drug plus 25 mL of EtOH 80%. The mixture was left under horizontal shaking at room temperature (25 °C) for 2 days, filtered, and extracted twice. Solutions were combined, concentrated under low pressure to eliminate EtOH, frozen (−24 °C), and lyophilized.

The 50% hydroalcoholic dried extract (50%HA) Axtragyl™ was purchased from Giellepi S.p.A. Health Science Division. The extract was reported to contain 30% maltodextrins as eccipients.

For the quantitative HPLC analysis, the following standards were used: Astragaloside IV, European Pharmacopoeia (EP) reference standard (97.8%) and formononetin ( ≥99% by HPLC) from Sigma-Aldrich. Dextrans with increasing and defined molecular weights (5000, 150000, 270000, 670000 Da) were from Sigma-Aldrich. The full characterization of the *Astragalus* extracts has been previously published^13^.

RETRACTED

Subsequently, 50%HA was fractioned using solvents with increasing polarity. The crude extract was suspended in water and extracted with 1) dichloromethane, 2) ethyl acetate and 3) butanol. Dried extracts were obtained by evaporation of dichloromethane, ethyl acetate and buthanol, using a rotary evaporator in vacuum under reduced pressure at 40 °C, or by freezing and lyophilization of the water fraction. The dried weight of the single fractions compared to the quantity of the total extract was: 1) dichloromethane fraction, 22%; 2) ethyl acetate fraction, 3%; 3) butanol fraction, 6%; 4) water fraction, 69%.

### Animals

Male Sprague-Dawley (SD) rats (Harlan, Varese, Italy) weighing approximately 200 to 250 g at the beginning of the experimental procedure were used. Pirc (F344/NTac-Apc^am1137^) rats, originally obtained from Taconic (Taconic Farms, Inc. USA) were bred in CESAL (University of Florence, Italy) in accordance with the Commission for Animal Experimentation of the Italian Ministry of Health (Femia *et al*.^44^). Animals were housed in CeSAL (Centro Stabulazione Animali da Laboratorio, University of Florence) and used at least 1 week after their arrival.

Four rats were housed per cage (size 26 × 41 cm) kept at 23 ± 1 °C with a 12 h light/dark cycle, light at 7 a.m; were fed a standard laboratory diet and tap water *ad libitum*. All animal manipulations were carried out according to the Directive 2010/63/EU of the European parliament and of the European Union council (22 September 2010) on the protection of animals used for scientific purposes. The ethical policy of the University of Florence complies with the Guide for the Care and Use of Laboratory Animals of the US National Institutes of Health (NIH Publication No. 85-23, revised 1996; University of Florence assurance number: A5278-01). Formal approval to conduct the experiments described was obtained from the Animal Subjects Review Board of the University of Florence. Experiments involving animals have been reported according to ARRIVE guidelines^51^. All efforts were made to minimize animal suffering and to reduce the number of animals used.

### Oxaliplatin model

SD rats were treated with 2.4 mg kg^−1^ oxaliplatin, administered i.p. for 5 consecutive days every week for 3 weeks (15 i.p. injections)^52^. Oxaliplatin was dissolved in 5% glucose solution.

RETRACTED

The model used for the present research is consistent with the clinical practice. The dose of 2.4 mg kg^−1^ oxaliplatin corresponds to the common human dosage (considering the Km factor 37 for the conversion of animal doses to the Human Equivalent Dose). The daily repeated administration of 2.4 mg kg^−1^ performed in the animal model provides a cumulative dose of 36 mg kg^−1^ corresponding to 1332 mg/m^2^. This dosage mimics the clinical cumulative oxaliplatin dose causing chronic neuropathy. The inorganic platinum plasmatic level on day 21 is 3.573 ± 0.217 μg/mL in our conditions, in line with human plasma concentrations^53^. Control animals received an equivalent volume of 5% glucose i.p. Behavioral and biochemical tests were performed on day 21. In the experiment with Pirc rats, 9 female Pirc rats, aged 8 months were randomly allocated to oxaliplatin treatment (n = 4) or to the same treatment with 50%HA (n = 5). Oxaliplatin treatments of Pirc rats were set up considering the higher sensitivity to oxaliplatin toxicity of these animals in comparison to SD rats. The dose of 1.5 mg kg^−1^ was injected i.p. twice a week for 4 weeks till the full development of painful neuropathy.

### Extract treatments

The extracts, Aqu, 20%HA and 50%HA, were suspended in 1% carboxy methyl cellulose (CMC) and administered p.o. every day for 3 weeks to SD rats. Aqu and 20%HA were administered at 300 mg kg^−1^ whereas 50%HA was administered in a dose range of 30 to 300 mg kg^−1^. The fractions obtained from 50%HA were administered as follows: 1) dichloromethane fraction, 66 mg kg^−1^; 2) ethyl acetate fraction, 9 mg kg^−1^; 3) butanol fraction, 18 mg kg^−1^; 4) water fraction, 207 mg kg^−1^. These doses were obtained considering the weight percent of the fractions (22%, 3%, 6% and 69% for fractions 1–4, respectively) compared to the quantity of the total extract and referred to the total extract dose of 300 mg kg^−1^. Extracts, or fractions, were orally administered every day for 3 weeks starting from the first day of oxaliplatin administration.

Pirc rats were treated with 300 mg kg^−1^ 50%HA p.o. daily for 4 weeks starting from the first day of oxaliplatin administration. Behavioral evaluations were performed 24 h after the last injection when not otherwise specified.

### Paw pressure test

The nociceptive threshold in the rat was determined by an analgesimeter (Ugo Basile, Varese, Italy) as previously described^19^ and reported in detail in the supplementary material (Supplementary Methods).

### Von Frey test

An electronic Von Frey hair unit (Ugo Basile, Varese, Italy) was used according to a previously described method^19^ and reported in detail in the supplementary material (Supplementary Methods).

RETRACTED

### Cold plate test

The Cold plate apparatus was used according to a previously described method^19^. The temperature of the cold plate was kept constant at 4 °C ± 1 °C. The method is reported in detail in the supplementary material (Supplementary Methods).

### Sciatic nerves examination

On day 21, at the end of the last behavioral test session, SD rats belonging to each group were sacrificed under general anesthesia and ipsilateral sciatic nerves were fixed, dehydrated and infiltrated with paraffin (Diapath, Milan, Italy). Sectioned tissues were evaluated immunohistochemically for p-NF-H as reported^19^. For details, see the supplementary material (Supplementary Methods).

### L4-L5 DRG examination

SD rat lumbar dorsal root ganglia were subjected to the treatment described for the sciatic nerves, sectioned, and stained using the Azan-Mallory method as previously reported^19^. The ATF-3 expression in L4-L5 DRGs was evidenced by the use of an anti-ATF-3 primary antisera (rabbit anti-ATF-3, 1:500; Santa Cruz Biotechnology), evidenced with diaminobenzidine as reported^19^. For details, see the supplementary material (Supplementary Methods).

### Immunohistochemistry of spinal cord and brain glia

On day 21, SD rats were sacrificed, the L4/L5 segments of the spinal cord were exposed from the lumbovertebral column via laminectomy and identified by tracing the dorsal roots from their respective DRG. The brains were removed, sliced in coronal sections and areas of interest were identified using Paxinos and Watson’s atlas (Paxinos and Watson, 1982). Quantification of the number and morphology of Iba1 immunoreactive microglia (rabbit, 1:1000; Wako Chemicals, Richmond, USA) and GFAP immunoreactive astrocytes (mouse, 1:5000; Chemicon, Temecula, USA) in the superficial dorsal horns of the spinal cord and in brain areas were performed in four cryostat sections (20 μm) by a previously reported method^19^,^21^. For details see the supplementary material (Supplementary Methods).

### mRNA level analysis

The sciatic nerve, L4-L5 DRGs and spinal cord of SD rats (day 21) were collected as described above. mRNA was extracted using TRI – Reagent© (Sigma Aldrich, Milan, Italy). cDNA was obtained using the iScript cDNA Synthesis Kit^®^ (Bio Rad, Milan, Italy) according to the manufacturer’s protocol. Nrf2 (Nuclear factor (erythroid-derived 2)-like 2) mRNA (GenBank accession number: NM_031789.2) was amplified using the following rat gene specific primers: forward: 5′ TGA CTC TGA CTC CGG CAT TTC 3′, reverse 5′ TCC ATT TCC GAG TCA CTG AAC 3′. NQO1 (NAD(P)H dehydrogenase, quinone 1) mRNA (GenBank accession number: NM_017000.3) was amplified using the following rat gene specific primers: forward: 5′ TCA TTT GGG CAA GTC CAT TCC 3′, reverse 5′ TGA GCA ATT CCC TCC TGC CCT 3′. 18 S ribosomal RNA (GenBank accession number: NR_046237.1) was considered as housekeeping gene and amplified using: forward: 5′ TAC CAC ATC CAA GGA AGG CAG CA 3′, reverse 5′ TGG AAT TAC CGC GGC TGC TGG CA 3′. Both sequences were amplified by GoTaq^®^ Flexi DNA Polymerase 2,500 U (Promega, Milan, Italy). The amplicons were electrophoresed in 1.8% agarose gel containing ethidium bromide. The resultant bands were then quantified by densitometry and the intensity of the signal normalized to18S, thus correcting for any possible uneven loading of RNA.

RETRACTED

### Liver and kidney histopathological examination

The liver and kidney (SD rats, day 21) were removed, cut into small pieces, and fixed in 10% neutral buffered formalin. After dehydration in gradual ethanol (50% to 100%), they were cleared in xylene and embedded in paraffin. Sections (5 μm thick) were stained with hematoxylin and eosin dye and observed under a light microscope at an original magnification of 20X and 40X.

### Determination of apoptosis in colon tumors and normal colon of Pirc rats

After the 4-week treatments (described above), apoptosis was evaluated in paraffin-embedded sections (4 μm thick) of normal colonic mucosa and tumors stained with hematoxylin-eosin, as reported^54^. At least 15 full longitudinal crypt sections of normal mucosa/rat were scored at the microscope, determining the presence of cells in each crypt with the following characteristics of apoptosis: cell shrinkage, loss of normal contact with the adjacent cells of the crypt, chromatin condensation or formation of round or oval nuclear fragments (“apoptotic bodies”). When clusters of more than one apoptotic body were seen within the diameter of one cell, these bodies were considered as fragments of one apoptotic cell. Tumor apoptosis was determined by scoring at least 500 cells/tumor for the presence of apoptotic cells that were coded as described above. In tumors and colon mucosa, apoptosis was scored by a single observer on coded samples and quantified as apoptotic index (AI = number of apoptotic cells/cells scored  × 100).

### Statistical analysis

Behavioral measurements were performed on 10 rats for each treatment carried out in 2 different experimental sets. Results were expressed as means ± S.E.M. and the analysis of variance was performed by one-way ANOVA. A Bonferroni’s significant difference procedure was used as post-hoc comparison. One-way ANOVA followed by Bonferroni post-test were used for the mRNA level analysis of comparisons between groups. Histologic, morphometric, and immunohistochemical analyses were performed on 6 rats per group, evaluating 6 sciatic nerves, 6 L4-L5 DRGs, and 6 spinal cord sections for each animal. DRG values are reported as means of L4 and L5. One-way repeated-measures analysis of variance followed by the Student-Newman-Keuls post hoc test was used to compare the percentage of ATF-3-positive neurons in small, medium, and large neurons in L4-L5 DRGs of oxaliplatin-treated rats. Histological studies of Pirc rats were analyzed by the t-test. For the rest of the comparisons, a Mann-Whitney test was used.

RETRACTED

In all experimental procedures, the investigators were blind to the experimental status of each animal. In addition, all images were captured and analyzed by an investigator other than the one who took measurements to avoid possible bias. Data were analyzed using the “Origin 9” software (OriginLab, Northampton, MA). Differences were considered significant at a *P* < 0.05.

## Additional Information

**How to cite this article**: Di Cesare Mannelli, L. *et al. Astragali radix:* could it be an adjuvant for oxaliplatin-induced neuropathy? *Sci. Rep.* **7**, 42021; doi: 10.1038/srep42021 (2017).

**Publisher's note:** Springer Nature remains neutral with regard to jurisdictional claims in published maps and institutional affiliations.

## Supplementary Material

Supplementary Information

## Figures and Tables

**Figure 1:** Behavioral measurements. (**A**) and (**B**) *Pain: mechanical noxious and non-noxious stimuli.* (**A**) Paw pressure test was used to measure sensitivity to a mechanical noxious stimulus. (**B**) The Von Frey test was used to measure the pain threshold as a response evoked by a non-noxious stimulus. (**C**) *Pain: thermal non-noxious stimuli*. The Cold plate test was used to evaluate the pain threshold measuring the latency to pain-related behavior (lifting or licking of the paw). Oxaliplatin (2.4 mg kg^−1^) was administered daily i.p. for 3 weeks. All *Astragalus* extracts (300 mg kg^−1^) were administered daily p.o. concomitantly with oxaliplatin. Behavioural evaluations were performed on day 21, 24 h after the last injection. Control animals were treated with vehicles. Each value represents the mean of 12 rats *per* group, performed in two different experimental sets. Values are represented as mean ± SEM. *P < 0.01 *versus* saline treatment; ^P < 0.05 and ^^P < 0.01 *versus* oxaliplatin treatment.

**Figure 2:** Behavioral measurements. *Pain: subchronic and acute effect of 50%HA.* On day 21, the pain reliever effect of 50%HA was evaluated by Paw pressure test. Oxaliplatin (2.4 mg kg^−1^) was injected daily i.p. for 3 weeks. (**A**) Increasing dosages (30, 100, 300 mg kg^−1^) of 50%HA were administered daily p.o., behavioural evaluations were performed 24 h after the last injection; (**B**) The acute effect of a single 50%HA administration (300 mg kg^−1^ p.o.) was evaluated 30 min after administration. Control animals were treated with vehicles. Each value represents the mean of 12 rats *per* group, performed in two different experimental sets. Values are represented as mean ± SEM. *P < 0.01 *versus* saline treatment; ^P < 0.05 and ^^P < 0.01 *versus* oxaliplatin treatment.

RETRACTED

**Figure 3:** Effect of 50%HA on oxaliplatin-dependent damages of the peripheral nervous system. The protective effect of 50%HA was evaluated on the sciatic nerve and in DRGs of treated animals on day 21. (**A**) *p-NF-H expression levels in sciatic nerve.* A representative immunohistochemical staining for p-NF-H in 10 μm longitudinal sciatic nerve sections is shown. For all images the scale bar = 10 μm and the original magnification was 20X. Bars show quantitative evaluation of neurofilament expression levels obtained by densitometric analysis. (**B**) *Morphological aspects of DRG nuclei and nucleoli.* The protective effect of repeated administrations of 50%HA was evaluated on oxaliplatin-damaged DRGs on day 21. Five μm DRG sections were stained by the Azan-Mallory method. Light micrographs (for all images: scale bar = 5 μm, original magnification 40X) were analyzed by measuring the occurrence of eccentric nucleoli (black arrowhead) and multinucleolated neurons (black arrow). Histograms show the incidence of nuclear and nucleolar pathological features in the absence (black bars) and in the presence of 50%HA (grey bars). (**C**) *ATF-3 expression in L4-L5 DRGs.* Typical immunohistochemistry images of ATF-3 expression in the DRG following oxaliplatin (oxaliplatin + vehicle) and oxaliplatin combined with 50%HA (oxaliplatin + 50%HA) treatments (day 21). ATF-3 staining is clearly punctuate and confined to the nucleus, shown as intense compact staining in brown (black arrows). The percentage of ATF-3-positive neurons in L4 and L5 DRGs is shown in the histogram. All images: scale bar = 10 μm, original magnification 20X. Each value represents the mean ± SEM of 6 rats *per* group, performed in two different experimental sets. *P < 0.05 *versus* vehicle + vehicle; ^*P* < 0.05 and ^^*P* < 0.01 *versus* oxaliplatin + vehicle.

**Figure 4:** Effect of 50%HA on oxaliplatin-dependent astrogliosis in the central nervous system (**A**) *Spinal cord.* On day 21, the number of GFAP-positive cells was measured in the dorsal horn of the spinal cord. Representative immunohistochemical staining is shown (scale bar = 10 μm and original magnification 20X, for all images) and black arrows evidenced that the activate astrocytic morphology induced by oxaliplatin administration (oxaliplatin + vehicle) is completely reverted by 50%HA presence. (**B**) and (**C**) *Brain areas.* The number of (**B**) GFAP- and (**C**) Iba-1-positive cells was evaluated in oxaliplatin-treated rats on day 21 analyzing the following areas: Cg1, cyngulate cortex area 1; S1, primary somatosensory cortex; M1, primary motor cortex; PAG, periaqueductal grey; mfb, medial forebrain bundle. Each value represents the mean ± SEM of 6 rats *per* group, performed in two different experimental sets. *P < 0.05 *versus* vehicle + vehicle; ^*P* < 0.05 *versus* oxaliplatin + vehicle.

RETRACTED

**Figure 5:** Histological evaluation of liver and kidney. (**A**) Effect of 50%HA on counteracting histopathological damages induced by oxaliplatin in the liver of rats. In the control animals (vehicle + vehicle), no liver damage was observed. Following oxaliplatin treatment (oxaliplatin + vehicle), fatty change (insert in oxaliplatin + vehicle, black arrows) and inflammatory cell with granular swelling were observed. The liver sections from oxaliplatin + 50%HA show little balloon changes in liver acinus, whereas 50%HA treated animals (vehicle + 50%HA) show no differences with control rats. Scale bar = 10 μm and original magnifications 20X for all the panels. (**B**) Effect of 50%HA on counteracting histopathological damages induced by oxaliplatin in the kidney of rats. The control animals (vehicle + vehicle) show any signs of kidney damage. Following oxaliplatin treatment (oxaliplatin + vehicle), kidney sections show glomerulopathy with Bowman’s space expansion (left panel, black asterisk), Bowman’s capsule thickening (left panel, black arrow), and mesangial expansion (left panel, black arrowhead), and tubule epithelium swelling and distension, together with severe vacuolar degeneration (right panel, black arrow). Oxaliplatin + 50%HA kidney section shows no pathological changes, as well as the kidney section from 50%HA-treated animals (vehicle + 50%HA). Scale bar = 10 μm and original magnifications 40X for all panels. All pathological observations were performed and graded by experienced and independent pathologists on 6 rats *per* group (two different experimental sets).

**Figure 6:** Pirc rats. (**A**) Pain threshold evaluation by Paw pressure test. Rats were treated with oxaliplatin 1.5 mg kg^−1^ i.p. twice a week for 4 weeks. 50%HA (300 mg kg^−1^) was administered p.o. daily for 4 weeks. Behavioural evaluations were performed 24 h after the last injection of both compounds. (**B**) Apoptotic index (number of apoptotic cells/cells scored x 100) in the normal mucosa (NM) and tumours from Pirc rats treated with oxaliplatin (oxaliplatin + vehicle) or oxaliplatin + 50%HA as explained in methods. Values are mean + SEM (n = 5, and 4 for NM and 9 and 13 for tumours in oxaliplatin + vehicle, and oxaliplatin + 50%HA, respectively). Bars with different superscript are significantly different (P < 0.01 with t-test).
